The article "How the COVID-19 Pandemic Impacted Oncological Molecular Diagnosis: A Picture from a National Reference Center for Molecular Pathology" was published in 2020. Journal: Biomed Res Int.

# How the COVID-19 Pandemic Impacted Oncological Molecular Diagnosis: A Picture from a National Reference Center for Molecular Pathology

**DOI:** 10.1155/2020/8397053

**Published:** 2020-10-01

**Authors:** Daniel Pinto, Luís Cirnes, Regina Pinto, Maria João Pina, Giancarlo Troncone, Fernando Schmitt

**Affiliations:** ^1^Serviço de Anatomia Patológica, Centro Hospitalar de Lisboa Ocidental, EPE, Lisboa, Portugal; ^2^NOVA Medical School, Lisboa, Portugal; ^3^IPATIMUP-Instituto de Patologia e Imunologia Molecular da Universidade do Porto/ I3S, Instituto de Investigação e Inovação em Saúde, University of Porto, Porto, Portugal; ^4^Escola Superior de Saúde, Instituto Politécnico do Porto, Porto, Portugal; ^5^Department of Public Health, University of Naples Federico II, Naples, Italy; ^6^Faculdade de Medicina da Universidade do Porto, Porto, Portugal

## Abstract

**Introduction:**

The Portuguese healthcare system had to adapt at short notice to the COVID-19 pandemic. We implemented workflow changes to our molecular pathology laboratory, a national reference center, to maximize safety and productivity. We assess the impact this situation had on our caseload and what conclusions can be drawn about the wider impact of the pandemic in oncological therapy in Portugal. *Material and Methods*. We reviewed our database for all oncological molecular tests requested between March and April of 2019 and 2020. For each case, we recorded age, sex, region of the country, requesting institution, sample type, testing method, and turnaround time (TAT). A comparison between years was made.

**Results:**

The total number of tests decreased from 421 in 2019 to 319 in 2020 (*p* = 0.0027). The greatest reduction was in clinical trial-related cases. Routine cases were similar between years (267 vs. 256). TAT was higher in 2019 (mean 15 days vs. 12.3 days; *p* = 0.0003). Medium- to large-sized public hospitals in the north of the country were mostly responsible for the reduction in cases (*p* = 0.0153).

**Conclusions:**

Case reduction was observed at hospitals that have mostly been involved in the treatment of COVID-19 and in the north of the country, the region worst-hit by the pandemic. Similar to other studies, our TAT decreased, even with a similar number of routine cases. Thus, we conclude that it is possible to successfully adapt the workflow of a molecular pathology laboratory to new safety standards without losing efficiency.

## 1. Introduction

On the second of March 2020, Portugal confirmed its first case of coronavirus disease 2019 (COVID-19) [1]. The number of infected rose rapidly, and by the end of April, there were more than 25,000 COVID-19 patients with nearly 1,000 people dead from the disease [2]. Although tragic, this scenario is far less severe than what was seen in other European countries, namely, Italy and Spain [3].

This might be explained in part by the swift measures taken by the Portuguese government, which implemented a state of emergency on the 18^th^ of March, merely a fortnight since the first confirmed cases and with a single confirmed death in the country. These measures included, amongst others, closing of schools and daycare, mandatory remote work, closing of all nonessential commerce and services, and confinement of most of the population to their residences, with a few exceptions [4].

It is of note that the impact of the disease in Portugal was heterogeneous, being felt with more intensity in the north of the country and, to a lesser degree, in Lisbon and surrounding areas [2].

Nationally, the government issued guidelines for a reorganization of the Portuguese National Health Service (PNHS) on the 16^th^ of March. As a result, all elective procedures and surgeries were suspended as resources were allocated to the treatment of COVID-19 patients. Oncological therapy was deemed the exception, however, and guidelines were emitted to enable continued therapy when safe conditions could be fulfilled and with reduced staff levels and other constraints related to the contingency programs [5, 6].

Our molecular laboratory (IPATIMUP, Porto) is a ISO15189-accredited laboratory and one of the national reference centers for molecular pathology in Portugal, handling samples from all over the country, from both public and private institutions [7–12].

During the COVID-19 outbreak, our laboratory kept performing predictive molecular testing on tissue (cytological and histological) and liquid biopsy samples. However, to better preserve the health and safety of our workers, in keeping with the 1-meter distance rule [13] and in an effort to minimize physical interactions between staff, some changes had to be made to our workflow: hands-on laboratory and clerk workers were divided in two teams of equal size, each rotating through the laboratory every 15 days; all staff allocated to the interpretation of molecular tests were placed in a regimen of remote working from home.

Given these constraints, we wondered what impact the current pandemic had in our case load of molecular tests and what conclusions could be drawn from this data about the impact of the COVID-19 pandemic on oncological therapy in Portugal. We also compared our results with a similar laboratory localized in Italy [13], a country most severely affected by the pandemic.

## 2. Materials and Methods

To monitor the impact of COVID-19 in the predictive oncologic molecular tests performed at our molecular laboratory, we reviewed our case database for all molecular tests requested between the period of March 16^th^ and April 15^th^ of 2019 and 2020, creating two separate cohorts. Only oncological somatic genomic tests were included in our analysis. Germinative genomic tests as well as tests for nonneoplastic diseases were excluded. Cases evaluated in the context of clinical trials, for which patient data was not available, were removed form age analysis but included in all others. Cases not signed out as of the time of writing were excluded from turnaround time (TAT) analysis but included in all others. The following variables were recorded for each case: age and sex, the region of the country from where the patient samples were received, whether the requesting institution was public or private, sample type, adopted testing methodologies, and turnaround time (TAT). In particular, TAT was considered the time between the receipts of samples to clinical reporting.

To analyze the provenance of the patients, we followed the Pathology National Hospital Reference Network guidelines, dividing the country into the following regions: north, center, Lisbon and Tejo Valley (LTV), and Algarve. According to the same document, national health service institutions were classified as either type I (containing basic and peripheral pathology laboratories), type II (containing intermediate level pathology laboratories), and type III (containing highly specialized pathology laboratories, located in central hospitals, academic, and oncological institutions) [14]. Private laboratories were grouped together under one category (PL).

Sample types were classified as either liquid biopsies (LB) or tissue/cytology material (TC), and the latter submitted either in paraffin blocks or glass slides. The following testing methodologies were used: next-generation sequencing (NGS), polymerase chain reaction- (PCR-) based capillary electrophoresis, Sanger sequencing, the Idylla^TM^ (Biocartis, Mechelen, Belgium) platform (fully automated real-time PCR), and digital PCR. NGS methodology in our laboratory mainly serves patients with lung cancer, some cases of CNS neoplasms, and cases of occult primary tumors, in search of actionable therapeutic targets. We use the oncomine FOCUS assay panel (Thermo Fisher Scientifics, Waltham, Massachusetts, USA). This panel includes 52 genes tested for a number of genomic alterations. Briefly, 35 genes are analyzed for hotspot mutations/insertion/deletion (in detail: *EGFR*, *BRAF*, *KRAS*, *NRAS*, *HER2*, *HER4*, *MET*, *PIK3CA*, and *ALK*); copy number variations (CNV) are evaluated for 19 genes, while gene fusion detection is covered for 23 genes, including *ALK*, *ROS1*, *KIF5B-RET*, *NTRK*, among others. This panel is run on Ion S5™ or S5 XL™ (Ion Torrent, Thermo Fisher, USA) with a minimum coverage of 500x and 2000x for DNA and RNA, respectively. Sanger sequencing in our laboratory is used in GIST tumors for *PDGFRA* and *C-KIT* genes, in some cases for BRAF in colon carcinomas and melanomas and PIK3CA in advanced breast carcinoma. In patients with clinical requests for the determination of microsatellite instability, a PCR (pentaplex) is performed and, after confirming that the amplification has occurred as expected, the PCR product run through clot analysis on the ABI3500 (Thermo Fisher, USA). The five monomorphic markers (BAT-26, BAT-25, NR-24, NR-21, and NR-27) are analyzed according to their standards. The fully automated real-time PCR (RT-PCR) platform Idylla^TM^ (Biocartis, Mechelen, Belgium) is used essentially for colon/rectal tumors in order to determine the status of *RAS* in routine cases as in clinical trials where our laboratory is the reference center. To obtain comprehensive information on clinically relevant mutational hotspots, two cartridges are sequentially employed in the following algorithm: *KRAS* cartridge first, moving on to *NRAS/BRAF* if *KRAS* mutations are not detected. When assays need to be highly sensitive, for example to detect T790M resistance mutation, Digital PCR by TaqMan probes on the 3D Digital system QuantStudio PCR System (Thermo Fisher Scientifics) is carried out. Preliminary to all abovementioned assays is the staff pathologist assurance that DNA/RNA is really extracted from viable tissue areas in which the tumor ratio is optimal, and the percentage of inflammatory cells and potentially amplification inhibitors (such as mucin and melanin) is minimal.

### 2.1. Statistical Analysis

A comparative analysis was done between the two cohorts regarding patient age, sex, sample size, distribution over time, region of provenance, type of institution, TAT, sample type, and exam type. Continuous variables were compared using the Mann-Whitney unpaired *t*-test, and discrete variables were compared using the Fisher or chi-squared tests, as appropriate. Statistical analysis was performed using the GraphPad Prism version 6.01 for Windows (GraphPad Software, La Jolla, California, USA, http://www.graphpad.com).

## 3. Results

### 3.1. Laboratory Workflow

The staff of the Molecular Laboratory of IPATIMUP is composed of 14 people with different skills, working full time at the laboratory (35 hours per week). From this total, five are fully dedicated to somatic genomic testing, including four biomedical assistants and one pathologist. During the COVID-19 outbreak, following the contingency plans of the institute, the director of the laboratory decided to divide the personnel in two teams shifting between *in loco* and remote work every fortnight. Each team was composed of six people, each including at least of two of the biomedical scientists dedicated to somatic testing. As mentioned, a pathologist working remotely supervised the processing of tissue samples. Interpretation of the results was done remotely using virtual private network (VPN) access over the internet to the computers in the laboratory. All staff were kept working full time, either *in loco* or remotely, to guarantee the adequate supply of reagents and to interpret the molecular testing results under the supervision of the chief biomedical scientist. Once per week, the whole team (both member working *in loco* and from home) had a virtual meeting to share progress reports and discuss quality and other relevant issues. All activities related to quality control were maintained in the same fashion.

### 3.2. Cohort Description

In 2019, during the period of March 16^th^ to April 15^th^, a total of 421 molecular tests were performed in our laboratory. From these, 80 were from nononcological samples and were excluded from analysis. This left us with 341 molecular tests performed on oncological cases. Of these, 74 were performed under clinical trial protocols and had no complete patient information. This left us with a total of 267 molecular tests with full data available for analysis.

In comparison, in the same period of 2020, a total of 319 molecular tests were performed in our laboratory, which is 102 less than the previous year (*p* = 0.0027). Interestingly, only 35 were from nononcological samples. The total of molecular tests carried out on oncological cases was 284. Similarly, to the number of nononcological samples, there was also a significant reduction in tests performed in the context of our clinical trial protocols, totaling only 28 in 2020. Since a further 10 cases were not signed out as of the time of writing, we were left with a total of 246 molecular tests with full data available for analysis in 2020.

A summary description of our cohorts can be found in Figure 1.

### 3.3. Demographics and Turnaround Time

In terms of demographics, from the 267 molecular tests with data available for demographic analysis performed in 2019, 103 (30.2%) belonged to female patients and 164 (48.1%) to male patients. The median age was 67 years (mean, 65.4 years; range, 0-89). From the 256 molecular tests with data available for demographic analysis performed in 2020, 101 (39.5%) belonged to female patients and 155 (60.5%) to male patients. The median age was 66 years (mean, 65.3 years; range, 36-94). The case distribution by age can be better appreciated in Figure 2. No statistically significant differences were found between the two cohorts with regard to age (*p* = 0.2070).

We calculated the TAT for each cohort. In 2019, the median TAT was of 15 days (mean, 14.8 days; range, 1-46), and in 2020, the median TAT was of 12 days (mean, 12.3 days; range, 2-42). A statistically significant difference was found between the two cohorts in terms of TAT (*p* = 0.0003). The TAT distribution can be seen in Figure 2.

### 3.4. Requesting Institutions and Geographical Differences

Special care was taken to assess the features of the institutions issuing fewer requests. Our data show that the overall decrease in testing is mostly due to the PNHS institutions (301 requests in 2019 vs. 236 requests in 2020). Interestingly though, whereas PNHS type I institutions (i.e., smaller regional hospitals) show an increase in both number and relative percentage of molecular tests requested [99 (29.03%) vs. 102 (35.92%)], PNS types II and III (i.e., medium to large hospitals and reference centers) featured a significant decrease in the number of tests requested [202 (59.2%) vs. 134 (47.2%)]. In fact, since the number of tests requested by private laboratories increased, the reduction in the number of requested tests comes solely from types II and III PNS institutions (*p* = 0.0153).

In terms of region, the largest decrease in testing comes from the Northern region of Portugal, encompassing all territory roughly from the Spanish border with Galiza down to the Douro river [165 (48.4%) vs. 129 (45.42%)]. The cases from LTV and Algarve also decreased, whereas the cases from the Center saw a slight increase (*p* = 0.0146).

These results can be seen in greater detail in Table 1.

### 3.5. Tissue and Cytology vs. Liquid Biopsies

Liquid biopsies are mostly done in our institution for the detection of EGFR T790M resistance mutations in the context of lung cancer. It is worth noting that although the absolute number of both sample types decreased, this was more evident in liquid biopsies. This difference in the distribution showed statistical significance (*p* = 0.0067).

### 3.6. Molecular Tests Performed

Comparing 2019 with 2020, we found a significant decrease in the number and proportion of Idylla^TM^ tests [145 (42.5%) vs. 80 (28.2%)], as well as an increase in the number of molecular tests performed by Sanger sequencing [29 (8.5%) vs. 38 (13.38%)] and PCR-based capillary electrophoresis [2 (0.6%) vs. 17 (6.0%)]. These differences are statistically significant (*p* < 0.0001). The remaining test types (digital PCR and NGS) were performed at similar levels between both years, with NGS showing a slight decrease in absolute numbers but a slight increase in preponderance. These results can better be appreciated in Table 1 and are schematized on Figure 3.

It is of note that the tests performed in the context of clinical trials are all done in the Idylla^TM^ platform check material and methods, and those decreased by a total of 46, year-on-year.

## 4. Discussion

The comparison between our two cohorts highlights the challenges that the Portuguese National Health System (PNHS) underwent during the first peak of the COVID-19 pandemic. In our series, there was a decrease in the absolute number of molecular tests. However, if we exclude those performed under clinical trial protocols, we can see that the difference between 2019 and 2020 is not that expressive (267 vs. 256 routine cases tested, respectively). In fact, both series seemed to be equivalent, at least in terms of age and sex distribution. Thus, it is not farfetched to conclude that no significant changes were observed in the volume of routine predictive molecular testing in our institution.

These results are similar to what was recently reported in an Italian reference center [13], where even during the COVID-19 outbreak, oncological patients were properly tested for targeted treatment, as usual. Conversely, while molecular testing is maintained, the traditional histopathology and cytopathology has during the same time period decreased in our (data not shown) and in other institutions [15].

Remarkably, our molecular laboratory adapted to the health emergency and implemented measures to limit virus transmission, focusing on maintaining adequate social distance between staff members [16, 17]. For this reason and to avoid unnecessary contamination or exposure of our technicians, we reduced our team by half and had teams rotate each 15 days. Despite the reduction in staff (approx. 50%), our TAT was significantly better in 2020, during the peak of the pandemic, compared with the same period of last year. This is particularly remarkable if we consider that the total reduction in case load was of only around 5%, which highlights the successful adaption of our molecular pathology laboratory to the new work rotation: similar numbers of routine cases were handled between the two periods, and the response times were actually faster. As the pandemic progresses and we become accustomed to this new workflow organization, it is conceivable that some, if not most, of these changes may be kept after the pandemic, resulting in similar or better patient care, a less crowded work environment, and better satisfaction with work life for our technicians.

In a similar study, Malapelle et al. [13] also showed a significant reduction of the TAT in the pandemic period. In that study, the main reason pointed out by the authors was the adoption and prioritization of a fully automated testing platform, which proved a valuable tool in ensuring accurate biomarker evaluation and sustainable laboratory activity.

In fact, the published literature regarding the adoption of the Idylla^TM^ platform [18–20] shows that the technical switch toward such a system allows for a reduction in working hours, which is a clear benefit during situations of greater constraints, like the COVID-19 pandemic. Because these techniques require less hands-on time, they allow for more social distancing and better safety risk management. There are some disadvantages in the adoption of fully automated systems, however: increased cost per patient in some types of cancer, as lung cancer does not detect all actionable mutations recommended; the need for validation with NGS in some cases; and a relative inflexibility of the platform—this approach cannot be adopted in situations where there is a need to analyze a large panel of genes, as in the case of lung cancer patients. [10]

Contrary to what has been reported by Malapelle et al. [13], we observed a decrease of the use of the Idylla^TM^ platform.

It is conceivable that Idylla^TM^ is clearly advantageous during the pandemic [13, 18–20], being fast and easy with minimal analysis or hands-on time. However, in our laboratory, many of the tests usually performed using this platform are carried out in the context of clinical trials, and these decreased significantly in number. Despite the reduced numbers of staff, we did not observe an increase in the use of Idylla^TM^ for routine cases. This may be explained by the fact that in our institution most of the cases analyzed are from lung cancer patients, followed by colon cancer and SNC tumors, making it nearly impossible to switch our routine from NGS.

Since molecular testing is based on formalin-fixed and paraffin-embedded (FFPE) tissue and fixed smears, the possibility that the SARS-CoV-2 virus was present in samples was minimal [21]. Conversely, liquid-based cytology may represent a potential source of transmission if fixatives with low alcohol concentrations (<70%) are used. Since we cannot control the fixation process upstream, we did not use this type of material for molecular analysis during the pandemic. Serum for liquid biopsy analysis is submitted fresh and may represent a potential source of transmission; thus, we significantly reduced this type of assay.

Moving to the perspective our data gives us for the country as a whole, we noticed changes in the numbers coming from different types of requesting institutions. On the one hand, we did not see a reduction in cases from private laboratories and in fact even observed a slight increase. This may be explained by the fact that the private health sector was only marginally involved in the treatment of COVID-19 patients in our country. In contrast, we did see a significant reduction in the number of cases from public hospitals. This is more evident in the most-specialized institutions (PNHS types II and III). During the pandemic, many of these became reference centers for COVID-19 patients who, in general, were not treated in community hospitals (which tendentially are classified as PNHS type I). In terms of region, it is interesting to note that the largest and most significant decrease in tests ordered comes from the north of the country where our laboratory is located (Porto). The north region was by far the worst-hit region in Portugal, with approximately 2.5× the number of cases of the second worst-hit region, LVT (14726 total cases in the north vs. 5815 total cases in LVT, as of April 30^th^) [2]. This raises the possibility that the impact of the pandemic on oncological management could have been worse if the number of cases had been significantly higher in the country.

In conclusion, our findings show that during the COVID-19 pandemic, the Portuguese health system was able to successfully adapt and maintain oncological therapy within reasonable levels, while locking down the country and changing hospital routine to face the new infectious disease. Our results also reinforce the findings of other studies [13, 15] that COVID-19 emergency is changing the way we practice not only histo- and cytopathology but also predictive molecular pathology. This activity is crucial to extend and improve the life expectancy and quality of our oncological patients, and it is possible to successfully adapt the workflow of a molecular pathology laboratory to new safety standards without losing efficiency during these exceptional times, using different strategies adapted to the reality at hand.

## Figures and Tables

**Figure 1:** Cohort description.

**Figure 2:** Distribution of patient age and turnaround time.

**Figure 3:** Percentage of molecular tests performed in 2019 vs. 2020.

**Table 1:** Comparison between discrete variables evaluated in both cohorts.

Evaluated variables	Type	2019 (*N*)	2019 (%)	2020 (*N*)	2020 (%)	*p* value
Institution	PNHS type I	99	29.03%	102	35.92%	0.0153
	PNHS type II	111	32.55%	66	23.24%	
	PNHS type III	91	26.69%	68	23.94%	
	PL	40	11.73%	48	16.90%	
Region	North	165	48.39%	129	45.42%	0.0146
	Center	39	11.44%	45	15.85%	
	LTV	122	35.78%	108	38.03%	
	Algarve	15	4.40%	2	0.70%	
Sample	LB	36	10.56%	13	4.58%	0.0067
	TCB	305	89.44%	271	95.42%	
Molecular test	NGS	164	48.09%	147	51.76%	<0.0001
	Sanger	29	8.50%	38	13.38%	
	Idylla	145	42.52%	80	28.17%	
	PCR-based capillary electrophoresis	2	0.59%	17	5.99%	
	Digital PCR	1	0.29%	2	0.70%	
